This article has been retracted.

# Analysis on Characteristics of Magnetic Resonance Imaging Image under Low-Rank Matrix Denoising Algorithm in the Diagnosis of Cerebral Aneurysm

**DOI:** 10.1155/2021/9751009

**Published:** 2021-11-15

**Authors:** Jun Li, Jin Li, Qin Hu

**Affiliations:** Department of Radiology, The Jingmen No.1 People's Hospital, Jingmen, 448000 Hubei, China

## Abstract

This study was to explore the effect of a low-rank matrix denoising (LRMD) algorithm based on the Gaussian mixture model (GMM) on magnetic resonance imaging (MRI) images of patients with cerebral aneurysm and to evaluate the practical value of the LRMD algorithm in the clinical diagnosis of cerebral aneurysm. In this study, the intracranial MRI data of 40 patients with cerebral aneurysm were selected to study the denoising effect of the low-rank matrix denoising algorithm based on the Gaussian mixture model on MRI images of cerebral aneurysm under the influence of Rice noise, to evaluate the PSNR value, SSIM value, and clarity of MRI images before and after denoising. The diagnostic accuracy of MRI images of cerebral aneurysms before and after denoising was compared. The results showed that after the low-rank matrix denoising algorithm based on the Gaussian mixture model, the PSNR, SSIM, and sharpness values of intracranial MRI images of 10 patients were significantly improved (*P* < 0.05), and the diagnostic accuracy of MRI images of cerebral aneurysm increased from 76.2 ± 5.6% to 93.1 ± 7.9%, which could diagnose cerebral aneurysm more accurately and quickly. In conclusion, the MRI images processed based on the low-rank matrix denoising algorithm under the Gaussian mixture model can effectively remove the interference of noise, improve the quality of MRI images, optimize the accuracy of MRI image diagnosis of patients with cerebral aneurysm, and shorten the average diagnosis time, which is worth promoting in the clinical diagnosis of patients with cerebral aneurysm.

## 1. Introduction

Cerebral aneurysm refers to the bulge or globular vascular sac formed on the vascular wall of the intracranial artery. The abnormally swollen part of the vascular wall causes vascular rupture under long-term impact pressure, which is more common in the internal carotid artery system. It will show different symptoms if the location of cerebral aneurysm, the size of the tumor, and the occurrence of rupture and hemorrhage of the tube wall are different. The symptoms include disturbance of consciousness, vomiting, sudden headache, epileptic seizure, and meningeal irritation under the influence of subarachnoid hemorrhage; nerve compression symptoms such as oculomotor nerve palsy, visual field defect, and diplopia due to the space-occupying effect; and paresthesia and hemiplegia caused by spasticity and cerebral ischemia [1–3].

Computer tomography (CT), MRI, and digital subtraction angiography (DSA) are commonly used in the clinical diagnosis of cerebral hemangioma [4]. In the clinical CT detection process, a large degree of error will be caused due to breathing, and the DSA examination is the gold standard for clinical detection of cerebral aneurysm. Its image quality is high, but it is an invasive examination and is expensive, and there is also the possibility of adverse reactions such as neurological deficits and vasospasm [5]. MRI is currently the only nonradiation hazard and noninvasive cerebrovascular imaging technology. It is more sensitive to the identification and diagnosis of intracranial cerebral aneurysm. It can display the structure of blood vessels without the use of radiographic contrast agents. It shows a high signal on the fluid-attenuated inversion recovery (FLAIR) sequence, so it has become one of the efficient ways to screen for unruptured intracranial aneurysms in high-risk groups of intracranial aneurysms. However, the spatial resolution of MRI images is lower than that of CT and DSA, and it is easily interfered with by artifacts and takes a long time to scan. It is not the best choice for emergency, critically ill patients, and claustrophobic patients, showing a higher false negative rate (FNR) [6].

A large number of studies have pointed out that the traditional MRI and transmission process will be interfered with by Rician noise, and effective denoising processing can improve the quality of MRI images, thereby enhancing the diagnostic efficiency. In recent years, there have been many reports on denoising algorithms for MRI images, including filtering method, nonlocal means (NLM), image block prior denoising algorithm, block-based piecewise linear estimation algorithm, GMM-based block likelihood logarithmic expectation algorithm, and low-rank matrix factorization (LRMF) algorithm based on image sparsity [7]. Among them, the method of increasing the effect of the LRMD algorithm by adding the variation regular term can be divided into the nuclear norm minimization (NNM) and the LRMF. LRMF refers to a specific data item that seeks a matrix that is infinitely close to a noisy image, that is, a real image that is infinitely approaching. It is known that LRMF is a nonconvex optimization method, while NNM is a convex optimization method. It is a method of solving the target matrix through the restriction of the kernel norm. It is an approximate convex optimization solution of LRMF, which can be obtained by convex relaxation of the nonconvex optimized LRMF [8].

In summary, the feasibility of the LRMD algorithm for MRI images has been confirmed, but there is no relevant report about its application in clinical MRI image diagnosis of cerebral hemangioma. Therefore, the denoising process of MRI images of the cerebral aneurysm has to be further optimized. Based on the currently known data related to GMM and LRMD algorithm for processing the MRI images [9], the MRI image data of confirmed cerebral aneurysm patients were selected to simulate the construction of the MRI images for intracranial cerebral hemangioma for the LRMD algorithm, which is based on GMM that combines block priors, gradient sparse priors, and image block self-similarity. It could guide the clustering of noise image blocks, increase the correlation among MRI image blocks, and maintain or enhance the MRI image block matrix. In order to improve the denoising effect of the LRMD algorithm, the differences in MRI sharpness of cerebral aneurysm patients before and after the denoising were compared. This study is aimed at evaluating the denoising effect of the LRMD algorithm on cerebral aneurysm MRI images and measuring the value of the algorithm in clinical MRI diagnosis of cerebral aneurysm, so as to provide a reference for the diagnosis and treatment of cerebral aneurysm.

## 2. Materials and Methods

### 2.1. Basic Information of Research Objects

The MRI data of 40 patients with cAN diagnosed in hospital from June 2019 to December 2020 were selected as the study subjects; all cAN patients were 24 males and 16 females, and the age range of the patients was 28-74 years; the mean age was 46.51 ± 5.89 years. The inclusion criteria for this study were as follows: (1) patients were diagnosed with cerebrovascular disease by clinical symptoms and pathology; (2) all patients' disease and physical indications met the requirements of MRI examination, and no contraindication to the examination was found; and (3) patients were fully informed of the experimental study and signed the consent form. Exclusion criteria were as follows: (1) patients who had already undergone treatment for cerebrovascular disease, (2) patients who were unsuitable for MRI examination, (3) patients with psychiatric disorders who were unable to perform or refused to cooperate with the experimental study, etc. All processes of this study have been approved by the Ethics Committee of the Hospital, and the subjects included in the study have signed the informed consent form.

### 2.2. Clustering of Cerebral Aneurysm MRI Images Based on GMM

The MRI images of different organs were similar, so it was hard to distinguish the image blocks using the similar interference signals of different structures in the intracranial MRI images of cerebral aneurysm patients [10]. Thus, the MRI images of intracranial cerebral hemangioma were performed with clustering based on GMM combined with the a priori method of noise-free MRI image blocks. Firstly, the MRI image was set as *S*, which was divided according to the structural similarity. Then, the division results (*n* image blocks) were merged into a set, namely, *PS* = (*P*_1_*S*, ⋯, *P*_*i*_*S*, ⋯, *P*_*n*_*S*). In this set, *P*_*i*_*S* represented the matrix corresponding to the first image block. If the image block, *PS* could be classified into *w* categories; then, the probability of the image block *P*_*i*_*S* could be expressed by GMM, which was given as follows:

(1) $$\begin{array}{c} p\left(P_{i}S\left|\Theta \right.\right)=\overset{H}{\underset{h=1}{\sum }}w_{h}p_{h}\left(P_{i}S\left|\mu_{h},\right.\underset{h}{\sum }\right). \end{array}$$

In equation (1) above, *H* represented the GMM contained *H* Gaussian classes, *h* represented the number of corresponding Gaussian category, *w* represented the weight, *μ* represented the mean value, ∑ referred to the covariance matrix, and Θ represented the set composing the mean value *μ*, covariance matrix ∑, and weight *w* of each Gaussian category. It could be expressed as Θ = (*μ*_1_, ⋯, *μ*_*h*_, ∑_1_, ⋯, ∑_*h*_, *w*_1_, ⋯, *t*_*h*_). In addition, *p*(*P*_*i*_*S*|*μ*_*h*,_∑_*h*_) referred to the probability density function of the *h*^th^ Gaussian category, which could be written as

(2) $$\begin{array}{c} p\left(P_{i}S\left|\mu_{h},\right.\underset{h}{\sum }\right)=c\cdot \exp\left(-\frac{1}{2}{\left(P_{i}S-\mu_{h}\right)}^{T}\overset{-1}{\underset{h}{\sum }}\left(P_{i}S-\mu_{h}\right)\right). \end{array}$$

In the equation above, *c* represented the normalization constant, and the negative exponent was to show the Mahalanobis distance for correlation between *P*_*i*_*S* and *μ*_*h*_. On this basis, the class label *D* = (*d*_1_, *d*_2_, ⋯, *d*_*h*_), *d*_*i*_ ∈ {1, 2, ⋯, *R*} was adopted to simplify the expression. *p*(*P*_*i*_*S*, *d*_*i*_ = *h*|Θ) indicated that under the GMM parameter set Θ, *P*_*i*_*S*(*i*, ⋯, *h*) was independent of *P*_*i*_*S*(*i*, *j*, = 1, ⋯, *h*, *i* ≠ *j*). In the GMM parameter set Θ, the probability of *PS* to cluster into category *R* was calculated with the below equation:

(3) $$\begin{array}{c} p\left(PS,D\left|\Theta \right.\right)=\overset{h}{\underset{i-1}{\prod }}p\left(P_{i}S,d_{i}\left|\Theta \right.\right). \end{array}$$

After taking the logarithm of both sides, equation (3) could be transferred as follows by combining with equation (2):

(4) $$\begin{array}{c} \overset{h}{\underset{i=1}{\sum }}\log p\left(d_{i}\right)p\left(P_{i}S\left|d_{i}\right.\right)=\overset{h}{\underset{i=1}{\sum }}\log w_{d_{i}}p_{d_{i}}\left(P_{i}S\left|\mu_{d_{i}},\underset{d_{i}}{\sum }\right.\right). \end{array}$$

The final clustering results of cerebral aneurysm MRI images based on GMM are shown in Figure 1.

### 2.3. Analysis of the Model Construction of Cerebral Aneurysm MRI Images Based on the LRMD Algorithm

The cerebral aneurysm MRI image *S* with a given noise was divided into blocks to obtain a set *P* = (*P*_1_*S*, *P*_*i*_*S*, ⋯, *P*_*h*_*S*). It is assumed that the GMM parameter set was known by learning the information of the noise-free MRI image block, *PS* could be divided into *H* categories based on the GMM prior. ${\bar{P}}_{a}X=\left[P_{h_{1}},\cdots ,P_{h_{d\left(h\right)}}\right]$ referred to the matrix composed of all image blocks (vectorization) in the *H*^th^ category, and *d*(*h*) represented the number of all similar image blocks in the *H*^th^ category. The image blocks in the same Gaussian class contained similar structural information, so ${\bar{P}}_{h}S$ could be decomposed into the below equation:

(5) $$\begin{array}{c} {\bar{P}}_{h}S=Q_{h}+T_{h}. \end{array}$$

In equation (5), *Q*_*h*_ referred to the low-rank matrix, *T*_*h*_ represented the noise matrix, and the low-rank matrix referred to the image data after denoising. It was assumed that the noise of each pixel of the image is independent and identically distributed; then, $p\left({\bar{P}}_{h}S\left|Q_{h}\right.\right)⟶\exp\left(1/\sigma^{2}{\left\|{\bar{P}}_{a}S-Q_{h}\right\|}_{V}^{2}\right)$ could be obtained from the perspective of conditional probability, and the energy function *E*(*Q*_*h*_) could be expressed as follows:

(6) $$\begin{array}{c} E\left(Q_{h}\right)=\tau {\left\|Q_{h}\right\|}_{*}+\frac{1}{\sigma^{2}}{\left\|{\bar{P}}_{h}S-Q_{h}\right\|}_{F}^{2}. \end{array}$$

In the equation above, *τ* referred to the normal number, *σ* represented the noise standard deviation, ‖‖_∗_ was the matrix kernel norm, and *F* was the matrix Frobenius norm. The rank minimization as shown in equation (6) could be optimized and solved by minimizing the weighted kernel norm. *W*∑*B*^*x*^ was determined as the SVD decomposition of ${\bar{P}}_{h}S$; then, equation (7) could be obtained:

(7) $$\begin{array}{c} {\hat{Q}}_{a}={WG}_{C}\left(\sum \right)H^{B}. \end{array}$$

In summary, for a given noisy MRI image *S*, the noise-free MRI image *S* could be reconstructed under the architecture of the noise-free MRI image prior (GMM prior) and the MRI image block self-similarity prior decomposition denoising model. The model equation was expressed as

(8) $$\begin{array}{c} \left(\hat{A},\hat{D},\left\{Q_{h}\right\}\right)=\underset{\hat{S},\hat{D},\left\{Q_{h}\right\}}{\arg\min}\frac{\lambda }{\sigma^{2}}\left\|S-A\right\|\begin{array}{c} 2\\ 2 \end{array}-\log p\left(PA,D\left|\Theta \right.\right)+\overset{h}{\underset{h-1}{\sum }}E\left(Q_{k}\right). \end{array}$$

The cerebral aneurysm detection process based on GMM prior and MRI image block self-similarity prior is shown in Figure 2.

### 2.4. Evaluation Indicators and Diagnosis Methods for Cerebral Aneurysm MRI Image Based on LRMD Algorithm

The impacts of LRMD algorithm processing on the quality of cerebral aneurysm MRI images were evaluated based on several different indicators, including mean square error (MSE), PSNR, and SSIM. MSE and PSNR described the error between the target image *z* and the original image *x* from the perspective of pixel value, while SSIM took into account the characteristics of the human visual system, which would make the evaluation results more consistent with the human senses.

MSE was an index that described the difference between the target image and the original image. The reference target image was supposed as *z*, the original image was set to *x*, and its size was *L* × *O*. The calculation equation of MSE was shown in equation (9), which showed the MSE of pixel value error between the target image and the original image at all the same coordinates (*x*, *y*):

(9) $$\begin{array}{c} \text{MSE}\left(z,x\right)=\frac{1}{LO}\overset{L}{\underset{i=1}{\sum }}\overset{O}{\underset{j=1}{\sum }}{\left(z\left(i,j\right)-x\left(i,j\right)\right)}^{2}. \end{array}$$

This indicator represented the error of the entire image. The smaller the MSE value, the higher the quality of the image to be evaluated and the closer it was to the ideal image. As the image size increased, the MSE value also increased, and the root mean square error (RMSE) expression was obtained by taking the square root of the MSE. The specific equation is shown in

(10) $$\begin{array}{c} \text{RMSE}\left(z,x\right)=\sqrt{\frac{1}{LO}\overset{L}{\underset{i=1}{\sum }}\overset{O}{\underset{j=1}{\sum }}{\left(z\left(i,j\right)-x\left(i,j\right)\right)}^{2}}. \end{array}$$

There was a correlation between PSNR and MSE, which could be expressed as follows:

(11) $$\begin{array}{c} \text{PSNR}\left(z,x\right)=10\log_{10}\left(\frac{G^{2}}{\text{MSE}\left(z,x\right)}\right). \end{array}$$

*G* in the above equation represented the peak signal. The *G* value 255 corresponding to the 8-bit grayscale image used in this study was applied to equation (11); then, equation (12) could be obtained:

(12) $$\begin{array}{c} \text{PSNR}\left(z,x\right)=10\log_{10}\left(\frac{255^{2}}{\text{MSE}\left(z,x\right)}\right). \end{array}$$

The above equation showed that the smaller the MSE, the greater the PSNR, and the closer the original image was to the target image, the better the quality.

SSIM indicated the degree of similarity between the target image *f* and the original image *g* in terms of brightness, contrast, and structure, so that the evaluation results were more in line with the human senses. The calculation equations for brightness, contrast, and structure contrast were shown in equations (13), (14), and (15), respectively:

(13) $$\begin{array}{c} L\left(z,x\right)=\frac{2\mu_{z}\mu_{x}+c_{1}}{{\mu^{2}}_{z}{\mu^{2}}_{x}+c_{1}}, \end{array}$$

(14) $$\begin{array}{c} C\left(z,x\right)=\frac{2\sigma_{z}\sigma_{x}+c_{2}}{{\sigma^{2}}_{z}{\sigma^{2}}_{x}+c_{2}}, \end{array}$$

(15) $$\begin{array}{c} S\left(z,x\right)=\frac{2\sigma_{zx}+c_{3}}{\sigma_{z}\sigma_{x}+c_{3}}. \end{array}$$

The calculation equation of SSIM that integrated the three factors (brightness, contrast, and structure) could be written as follows:

(16) $$\begin{array}{c} \text{SSIM}\left(z,x\right)=\left(L{\left(z,x\right)}^{\alpha }\cdot C{\left(z,x\right)}^{\beta }\cdot S{\left(z,x\right)}^{\gamma }\right). \end{array}$$

In the equations above, *μ*_*z*_, *μ*_*x*_, *σ*_*z*_, and *σ*_*x*_ represent the mean values and standard deviations of the target image *z* and the original image *x*, respectively; *σ*_*zx*_ was the covariance of *z* and *x*. The sum of *c*_1_ = (*h*_1_*P*)^2^, *c*_2_ = (*h*_2_*P*)^2^, and *c*_1_ = *c*_2_/2 was constants, where *P* was the pixel value range of the MRI image. According to experience, if *h*_1_ = 0.01 and *h*_2_ = 0.03, and when *α* = *β* = *γ* = 1, SSIM, ∈[0, 1] approached 1, the original image *x* and the target image *z* were very similar, and the quality of image *x* was higher.

### 2.5. Evaluation of MRI Diagnostic Effect of Cerebral Aneurysm

In this study, the impact of the low-rank matrix denoising algorithm with Gaussian mixture model on the diagnostic efficiency of MRI images of cerebral aneurysms was comprehensively evaluated by comparing the average diagnostic time and diagnostic accuracy of MRI images of patients with cerebral aneurysms before and after processing by the low-rank matrix denoising algorithm with Gaussian mixture model.

### 2.6. Statistical Methods

The test data was processed using SPSS19.0 statistical software. The mean ± standard deviation$\left(\bar{x}\pm s\right)$ was adopted to express the measurement data. The comparison of the means of each group was performed by *t*-test. The count data was given in the form of percentage (%), and the *χ*^2^ test was adopted. *P* < 0.05 indicated that the difference was statistically significant.

## 3. Results

### 3.1. Comparison on Quality Indicators of Cerebral Aneurysm MRI Images under Different Noise Intensities

The analysis results on the MRI image quality indicators of cerebral aneurysm patients showed that under the same noise intensity, the difference in PSNR under different *K* values was very small (as illustrated in Figure 3).  Figure 4 reveals that with the increase of the noise intensity, the RMSE continued to rise, indicating that the greater the noise intensity, the lower the similarity between the MRI image and the original image.

### 3.2. Quality Evaluation of MEI Image Processed by GMM-Based LRMD Algorithm

The PSNR scores of MRI images processed based on Gaussian mixed low-rank matrix denoising algorithm were compared with those of MRI images before processing (Figure 5), and the results showed that before MRI image denoising, the PSNR scores of MRI images were 40.01, 30.12, and 26.07 under the conditions of 1%, 3%, and 5% noise levels, respectively, while after the Gaussian mixed low-rank matrix denoising algorithm processing, the PSNR scores of MRI images became 45.02, 38.15, and 35.07 under the conditions of 1%, 3%, and 5% noise levels, respectively. The PSNR scores of MRI images were 45.02, 38.15, and 35.21 at 1%, 3%, and 5% noise levels, respectively, after processing with the Gaussian mixed low-rank matrix denoising algorithm, and the PSNR scores were significantly higher than those before denoising. The closer the denoised MRI images were to the original images, the higher the quality was, and the easier it was to diagnose cerebral hemangioma.

Figure 6 shows the comparison of SSIM values of MRI images before and after processing by the low-rank matrix denoising algorithm; from the figure, before MRI image denoising, the SSIM scores of MRI images were 0.89, 0.78, and 0.67 under the noise level of 1%, 3%, and 5% conditions, respectively, while after processing by the Gaussian mixed low-rank matrix denoising algorithm, based on the Gaussian mixed low-rank matrix denoising algorithm, the SSIM scores of MRI images became 0.99, 0.97, and 0.95 under 1%, 3%, and 5% noise level conditions, with significant differences between the two groups of data, and the PSNR scores all showed a significant upward trend compared with those before denoising, with statistical significance (*P* < 0.05). The lower the noise level, the closer the SSIM value was to 1 after denoising, which indicated that the similarity between the original image and the target image was higher, i.e., the image quality of the original image was higher.

### 3.3. Changes on MRI Image Characteristics of Cerebral Aneurysm Patients before and after the Processing by GMM-Based LRMD Algorithm

Figure 7 shows the MRI image features of the patient with cerebral aneurysm extracted before and after denoising by the Gaussian mixed low-rank matrix. The orange part of the figure was the image of the focal area of cerebral aneurysm in the MRI image of the patient extracted before and after the denoising process. Compared with the MRI image of the patient before denoising, the MRI image after denoising was obviously clearer in texture and the imaging of cerebral vascular aneurysm was also more obvious. In Figure 8, in terms of the clarity of the same MRI of the same patient, the image with 5% noise was less clear compared to the MRI image with 1% noise, and the denoising process could significantly change the visual clarity of the MRI image.

### 3.4. Diagnostic Accuracy and Average Diagnosis Time of MRI Images of Patients with Cerebral Aneurysm

Figure 9 shows the diagnostic accuracy and average diagnostic time of MRI images of patients with cerebral aneurysm before and after processing by the low-rank matrix denoising algorithm.  Figure 9(a) shows the diagnostic accuracy of MRI images of patients with cerebral aneurysm before and after the denoising process, and Figure 9(b) shows the average diagnostic time of MRI images of patients with cerebral aneurysm before and after the denoising process. The diagnostic accuracy of MRI images of patients with cerebral aneurysm increased from 76.2 ± 5.6% before denoising to 93.1 ± 7.9% after denoising, with a statistically significant difference (*P* < 0.05), while the average diagnostic time decreased from 28.7 ± 4.4 min to 10.2 ± 3.2 min, with a statistically significant difference (*P* < 0.05).

## 4. Discussion

MRI has features that allow accurate localization of lesions, acquisition of multidirectional imaging of tissues and organs, observation of cerebrovascular network distribution, etc., and is currently an important marker for the diagnosis of intracranial aneurysms [11, 12]. MRI is susceptible to Rician noise pollution during imaging or transmission. Therefore, the research of its denoising algorithm is of great significance and value for obtaining high-quality MRI. Currently, there are many related reports on MRI image denoising algorithms. Veraart et al. [13] constructed a denoising model based on random matrix theory in 2016. Klosowski and Frahm [14] conducted a review of the current status of MRI image denoising in 2017. Zhang et al. [15] confirmed the value of the MRI image denoising algorithm based on chi-squared unbias theory in clinical diagnosis in 2019. Huang and Lin [16] improved the evaluation parameters of MRI images. de Senneville et al. [17] proposed an iterative back-projection denoising algorithm for abdominal MRI in 2020. Recently, Moeller et al. [18] put forward new research progress regarding the nonparameter local low-rank denoising of dMRI images, and a major breakthrough was made in 4D stream MRI image denoising for cerebral aneurysm [19, 20]. It is an urgent clinical task to study how to upgrade the algorithm to complete the effective denoising of MRI images. The advancement of key technologies will bring good news to the clinical diagnosis and treatment of more diseases. The GMM-based LRMD algorithm was applied to the diagnosis of MRI images of cerebral aneurysm patients in this study to evaluate its impacts on the diagnostic efficiency of MRI images. The results proved that the algorithm could visibly improve the noise pollution of MRI images, enhance the overall sharpness of the image, and make the structure and texture in the image more obvious, thereby improving the diagnostic efficiency of cerebral aneurysm patients and reducing the FNR. However, when the image noise intensity was large, more noise residues would appear in the denoised images processed by this algorithm, so improvement of which had to be further studied.

## 5. Conclusion

In this study, the GMM-based LRMD algorithm was adopted to construct a brain image block algorithm and applied to the MRI image analysis and diagnosis of cerebral aneurysm patients, so as to explore the value of MRI processed by the GMM-based LRMD algorithm in the diagnosis of cerebral aneurysm. The results showed that the denoising degree of MRI images processed by the GMM-based LRMD algorithm was increased dramatically, and the image quality was greatly improved, which increased the diagnosis accuracy and efficiency of cerebral aneurysm. However, there are some shortcomings in this study; for example, the denoising process in this study will smooth out some detailed texture information to a certain extent, causing a certain degree of diagnostic error, and the low-rank matrix denoising algorithm based on the Gaussian mixture model in this study is currently used for MRI 2D images and will be further explored for 3D images in future work. In summary, the GMM-based LRMD algorithm for MRI images can greatly improve the quality of MRI images and provide a reference for the clinical diagnosis and treatment of cerebral aneurysm patients.

## Figures and Tables

**Figure 1:** Clustering results of cerebral aneurysm MRI images based on GMM. Note: (a–f) showed the image with 10% noise, the clustering result of noisy images, the clustering results of the iteration generation, the clustering results of the iteration 3 generations, the clustering results of the iteration 6 generations, and the image after denoising, respectively.

**Figure 2:** Clustering process of cerebral aneurysm MRI images based on GMM.

**Figure 3:** Comparison of denoising results under different noise intensities (*K* values).

**Figure 4:** RMSE under different noise intensities.

**Figure 5:** Comparison of PSNR scores before and after denoising. Note: ∗ indicated that the difference was visible in contrast to the value before denoising (*P* < 0.05).

**Figure 6:** Comparison of SSIM score of MRI image before and after the denoising. Note: ∗ indicated the difference was visible in contrast to the value before denoising (*P* < 0.05).

**Figure 7:** Comparison of MRI images of patients with intracranial cerebral hemangioma before and after processing by GMM-based LRMD algorithm. Note: the left image was the one before denoising, and the right image was the one after denoising.

**Figure 8:** Comparison of MRI images of patients with intracranial cerebral hemangioma under different noise intensities. Note: (a–c) shows the MRI images with 5% noise, 1% noise, and 0% noise, respectively. (d–f) Showed the redundant images of corresponding images (a–c), respectively.

**Figure 9:** Comparison of diagnostic accuracy and average diagnosis time of MRI images of patients with cerebral aneurysm before and after denoising processing.

## Data Availability

The data used to support the findings of this study are available from the corresponding author upon request.
